The article "miR-196a-2 Promotes Malignant Progression of Thyroid Carcinoma by Targeting NRXN1" was retracted in 2023. Reasons: signs of a paper mill; suspected computer-generated content; unreliable results or conclusions; concerns about the data.

# miR-196a-2 Promotes Malignant Progression of Thyroid Carcinoma by Targeting NRXN1

**DOI:** 10.1155/2021/4856820

**Published:** 2021-05-31

**Authors:** Yaohua Fan, MingJian Fei, Yan Li, Zhenzhen Gao, Yuzhang Zhu, Guiping Dai, Dongjuan Wu

**Affiliations:** ^1^Department of Oncology, The Second Affiliated Hospital of Jiaxing University, Jiaxing, Zhejiang Province 314000, China; ^2^Department of Pathology, The Second Affiliated Hospital of Jiaxing University, Jiaxing, Zhejiang Province 314000, China

## Abstract

Thyroid cancer (TC) is the most common endocrine malignant disease with a rising morbidity year by year. Accumulating studies have shown that microRNAs (miRNAs) play a regulatory role in the progression of various tumors, but the molecular regulatory mechanism of miR-196a-2 in TC is still unknown. qRT-PCR was employed to measure the expression of miR-196a-2 and NRXN1 mRNA in TC cells, while western blot was used to detect the protein expression of NRXN1. CCK-8, colony formation and flow cytometry assays were used to measure cell proliferation and apoptosis of TC cells. Dual-luciferase reporter gene assay was used to predict and verify the targeted binding relationship between miR-196a-2 and NRXN1. Our study results manifested that miR-196a-2 was dramatically overexpressed in cells of TC, while NRXN1 was lowly expressed. miR-196a-2 could promote cell proliferation and inhibit cell apoptosis of TC. Additionally, miR-196a-2 could also target and inhibit the expression of NRXN1. Silencing NRXN1 could reverse the inhibitory effect of miR-196a-2 downregulation on cell proliferation of TC, as well as the promoting effect on cell apoptosis. In a conclusion, we found that miR-196a-2 could promote cell proliferation and inhibit cell apoptosis of TC by targeting NRXN1. Therefore, miR-196a-2/NRXN1 is potential to be a molecular therapeutic target for TC.

## 1. Introduction

Thyroid cancer (TC) is mainly caused by canceration in thyroid nodules, and its incidence accounts for 2.5% of all cancers and about 90% of endocrine tumors [1]. According to statistics, the detection rate of TC has been increasing at an annual rate of 4.5% in recent years [2], which has seriously affected human health. The current treatments for TC mainly include surgery, radiotherapy, and chemotherapy. Although great progress has been made in these treatments, the outcome of patients with tumor recurrence and metastasis is still unsatisfactory, and the annual survival rate is only 59% [3, 4]. Therefore, it is essential to unveil underlying mechanism and pathogenesis of TC progression, thus providing us with a complete and advanced TC therapeutic regimen.

MicroRNAs (miRNAs) are a class of noncoding small RNA molecules that can bind to the complementary regions of mRNAs to regulate mRNA degradation or translation [5, 6]. Evidence existed that numerous miRNAs are aberrantly expressed in TC tissue, and they are pivotal in tumor pathogenesis. For example, Wang et al. indicated that miR-497 is downregulated in TC and miR-497 can inhibit growth and metastasis of TC by targeting brain-derived neurotrophic factor (BDNF) [7]. Zhao et al. also disclosed that miR-96-3p is upregulated in TC, and that miR-96-3p can directly target succinate dehydrogenase complex iron-sulfur subunit B (SDHB) to promote tumor metastasis [8]. Wu et al. [9] found that miR-429 restrains cell growth and induces apoptosis of human TC cells via targeting zinc finger E-box-binding homeobox 1 (ZEB1). Fu et al. [10] found that miR-196a-2 is upregulated in TC and serves as an independent adverse prognostic factor for TC. Tang et al. [11] found that miR-196a-2 is negatively correlated with overall survival of patients with TC. Thus, whether miR-196a-2 exerts a role in TC progression and how it functions need to be validated. In this study, the expression of miR-196a-2 in TC was determined and the effects of miR-196a-2 on cell proliferation and apoptosis were observed. Besides, the molecular mechanism of miR-196a-2 in TC was studied to finally furnish a theoretical basis for miR-196a-2 as a molecular therapeutic target for TC.

The article "miR-196a-2 Promotes Malignant Progression of Thyroid Carcinoma by Targeting NRXN1" was retracted in 2023. Reasons: signs of a paper mill; suspected computer-generated content; unreliable results or conclusions; concerns about the data.

## 2. Materials and Methods

### 2.1. Cell Culture

The three human TC cell lines are TPC-1 (BNCC338689), KTC-1 (BNCC340144), and FTC-133 (BNCC337959), and the normal human thyroid cell line is HTori-3 (BNCC338687). HTori-3 and KTC-1 cell lines were cultured in F-12k medium (BNCC341829). FTC-133 cell line was cultured in Roswell Park Memorial Institute 1640 (RPMI-1640) medium. TPC-1 cell line was cultured in L-15 (BNCC341687) medium. All mediums were supplemented with 10% fetal bovine serum (FBS). Cells were cultured in a humidified incubator with 5% CO_2_ at 37°C. All cell lines and medium were purchased from Bena Culture Collection (BNCC) (China).

### 2.2. Cell Transfection

miR-196a-2-mimic (miR-mimic), miR-196a-2-inhibitor (miR-inhibitor), sh-NRXN1, and their corresponding negative controls (NC-mimic, NC-inhibitor, and sh-NC) were all accessed from GeneChem (Shanghai, China). Lipofectamine 2000 (Invitrogen, Carlsbad, USA) at 50 nM was utilized to transfect miR-mimic, miR-inhibitor, sh-NRXN1, and their corresponding NC into TC cell FTC-133. After 48 h of transfection, cells were collected for follow-up studies.

### 2.3. Real-Time Quantitative Polymerase Chain Reaction (qRT-PCR)

Total RNA of cells was isolated according to the instructions of TRIzol reagent (Invitrogen, Thermo Fisher Scientific, Inc.). Complementary DNA (cDNA) was synthesized with the TransScript First-Strand cDNA Synthesis SuperMix Kit (TransGen Biotech, Beijing, China) following the protocol. Finally, qRT-PCR was performed on the Applied Biosystems 7500 detection system using TransStart Green qPCR SuperMix (TransGen Biotech, Beijing, China) per manufacturer's instructions. The relative expression was normalized by 2^-*ΔΔ*Ct^ method, with U6 and GAPDH applied as internal references for miR-196a-2 and NRXN1, respectively. The experiment was repeated three times. The primer sequences were detailed in Table 1.

The article "miR-196a-2 Promotes Malignant Progression of Thyroid Carcinoma by Targeting NRXN1" was retracted in 2023. Reasons: signs of a paper mill; suspected computer-generated content; unreliable results or conclusions; concerns about the data.

### 2.4. Western Blot

Cells were lysed with RIPA lysis buffer (Thermo Fisher Scientific, MA, USA) on ice for 10 min to obtain total proteins, and the protein concentration was quantified by BCA kit (Thermo Fisher, Waltham, USA). Thereafter, 30 *μ*g of protein samples was treated by sodium dodecyl sulfate-polyacrylamide gel electrophoresis (SDS-PAGE) for 90 min, with the separated proteins sequentially loaded on polyvinylidene fluoride (PVDF) membranes (Santa Cruz Biotechnology, Inc., USA). After blocked in 5% skim milk for 60 min, the membranes were incubated with primary antibodies rabbit anti-human NRXN1 or rabbit anti-human GAPDH overnight at 4°C, followed by addition of horseradish peroxidase- (HRP-) conjugated secondary antibody goat anti-rabbit IgG H&L for 1 h of hybridization at room temperature. Finally, ECL kit (Solarbio, Beijing, China) was used to detect the protein signals on the membranes according to the instructions. All antibodies used in this study were obtained from Abcam (Cambridge, UK). The experiment was repeated in triplicate.

### 2.5. Cell Counting Kit-8 (CCK-8) Assay

CCK-8 assay was employed to assess the proliferative ability of TC cell FTC-133. 100 μl of FTC-133 cells (2 × 10^4^ cells/ml) was inoculated into a 96-well plate, and then, the plate was arranged in a humidified incubator with 5% CO_2_ at 37°C for 0, 24, 48, and 72 h. At specified time point, 10 μl of CCK-8 reagent (Dojindo Molecular Technologies, Inc., Kumamoto, Japan) was provided for cell incubation at 37°C for 2 h. Finally, the optical density (OD) value of each well was tested at 450 nm by a microplate reader (Model 550; Bio-Rad Laboratories, Inc., Hercules, CA, USA). Each experiment was repeated three times.

### 2.6. Colony Formation Assay

To perform a colony formation assay, FTC-133 cells (4 × 10^2^) were inoculated into a 6-well plate, and the 6-well plate was placed in an incubator with 5% CO_2_ at 37°C for cell culture. The medium in the wells was replaced every 4 days and was discarded after visible colonies appeared. The colonies were fixed with 4% paraformaldehyde for 15 min at room temperature, followed by staining with 0.1% crystal violet at room temperature for 10 min. Afterwards, the residual crystal violet in the wells was washed away with PBS, and the number of colonies formed in the wells was counted. The experiment was repeated three times.

The article "miR-196a-2 Promotes Malignant Progression of Thyroid Carcinoma by Targeting NRXN1" was retracted in 2023. Reasons: signs of a paper mill; suspected computer-generated content; unreliable results or conclusions; concerns about the data.

### 2.7. Cell Apoptosis Assay

Apoptosis experiment was used to observe the apoptotic rate of TC cell FTC-133. First of all, 2 ml of FTC-133 cells (1 × 10^5^ cells/ml) was seeded in a 6-well plate and then cultivated in a humidified environment with 5% CO_2_ at 37°C for 24 h. Then, the cells were subjected to fluorescence staining according to the instructions of the FITC Annexin V Apoptosis Detection Kit (BD Biosciences, Franklin Lakes, NJ, USA), and FACS Caliber (BD Biosciences, Franklin Lakes, NJ, USA) was used to detect the cell apoptosis. The experiment was repeated three times: Q1 (mechanically dead cells (%)), Q2 (late apoptosis cells (%)), Q3 (early apoptosis cells (%)), and Q4 (live cells (%)). The formula is as follows: apoptosis rate = (Q2 + Q3)/(Q2 + Q3 + Q4).

### 2.8. Dual-Luciferase Reporter Gene Assay

For dual-luciferase detection, amplified mutant-type or wild-type NRXN1 3′-UTR (NRXN1-Mut or NRXN1-Wt) was cloned into the psiCHECK-2 dual-luciferase vectors (Promega, Madison, WI). Before transfection, 100 μl of TC cell FTC-133 (1.5 × 10^5^ cells/ml) was inoculated into a 96-well plate, and then, NRXN1-Mut/NRXN1-Wt and miR-mimic/NC-mimic were cotransfected into FTC-133 cells using Lipofectamine 2000 (Invitrogen; Thermo Fisher Scientific, Inc.). Forty-eight hours later, Firefly and Renilla luciferase activities were measured by the luciferase reporter analysis system (Promega, USA), and the experiment was repeated three times.

### 2.9. Statistical Analysis

Data management and analysis were processed by GraphPad Prism 6 (GraphPad Software Inc., San Diego, CA, USA). Measurement data were presented as mean ± standard deviation. The difference among multiple groups was assessed by one-way analysis of variance (ANOVA) for significance test, and then, the Student *t*-test was used for post hoc testing. Comparison between two groups was by Student's *t*-test for significance test. *P* < 0.05 was considered statistically significant.

## 3. Results

### 3.1. miR-196a-2 Is Upregulated in TC Cells

Accumulating references indicated that miRNAs play a vital regulatory role in various tumor progression. Combining relevant references, we chose miR-196a-2 that was rarely reported as the research object in this study. qRT-PCR was applied to observe miR-196a-2 expression level in normal thyroid epithelial cell HTori-3 and TC cells FTC-133, TPC-1, and KTC-1. It was found that miR-196a-2 expression was significantly higher in TC cells than that in HTori-3 cells, and the expression differences were the most significant in FTC-133 cells (Figure 1(a)). Therefore, FTC-133 cells were selected for the subsequent experiments. The above experiments illuminated that miR-196a-2 was highly expressed in TC cells.

The article "miR-196a-2 Promotes Malignant Progression of Thyroid Carcinoma by Targeting NRXN1" was retracted in 2023. Reasons: signs of a paper mill; suspected computer-generated content; unreliable results or conclusions; concerns about the data.

### 3.2. Silencing miR-196a-2 Restrains Cell Proliferation and Promotes Cell Apoptosis of TC

To further verify that miR-196a-2 could promote the malignant progression of TC, miR-inhibitor was firstly transfected into TC cell FTC-133, and it was confirmed by qRT-PCR that transfection of miR-inhibitor could downregulate miR-196a-2 expression in FTC-133 cells (Figure 2(a)). Then, the effect of silenced miR-196a-2 on the proliferation and apoptosis of FTC-133 cells was observed via cell biological functional experiments. The results of CCK-8 and colony formation assays presented that silencing miR-196a-2 could pronouncedly inhibit the proliferative and colony forming abilities of FTC-133 cells (Figures 2(b) and 2(c)). It was also turned out that silencing miR-196a-2 could significantly promote cell apoptosis of FTC-133 as evidenced by flow cytometry (Figure 2(d)). Through the above experiments, it was found that miR-196a-2 could promote cell proliferation and reduce cell apoptosis of TC.

### 3.3. NRXN1 Is the Direct Target of miR-196a-2

To further study the mechanism of miR-196a-2 promoting the malignant progression of TC, NRXN1 with targeted binding sites of miR-196a-2 was finally discovered (Figure 3(a)). To confirm the regulatory relationship between miR-196a-2 and NRXN1, the expression of NRXN1 in cells was firstly detected. The results demonstrated that the expression of NRXN1 in TC was markedly downregulated (Figures 3(b) and 3(c)). Next, the expression of NRXN1 in FTC-133 cells with silenced miR-196a-2 was assessed through qRT-PCR and western blot. The results presented that silencing miR-196a-2 dramatically upregulated the expression of NRXN1 in FTC-133 cells (Figures 3(d) and 3(e)). Finally, the targeted binding relationship between miR-196a-2 and NRXN1 was validated by dual-luciferase reporter gene assay. The results manifested that miR-196a-2-mimic would not affect the luciferase activity of the NRXN1-Mut group, but it would decrease the luciferase activity of the NRXN1-Wt group (Figure 3(f)). Based on the above studies, it was affirmed that miR-196a-2 could directly regulate the expression of NRXN1.

### 3.4. miR-196a-2 Regulates Cell Proliferation and Apoptosis of TC by Targeting NRXN1

To further confirm that miR-196a-2 promotes the malignant progression of TC by targeting NRXN1, NC-inhibitor+sh-NC, miR-inhibitor+sh-NC, and miR-inhibitor+sh-NRXN1 were transfected into FTC-133 cells, respectively. Then, qRT-PCR and western blot were employed to detect the expression of NRXN1 in FTC-133 cells in each group. The results appeared that the expression of NRXN1 was significantly downregulated in cells transfected with miR-inhibitor and sh-NRXN1 compared with that in cells transfected with miR-inhibitor alone (Figure 4(a)). Then, cell biological functional experiments were used to observe cell proliferation and apoptosis. The results of CCK-8 assay and colony formation assay revealed that the inhibitory effect of miR-inhibitor on cell viability and colony formation of TC could be reversed by sh-NRXN1 (Figures 4(b) and 4(c)). Apoptosis assay also demonstrated that sh-NRXN1 reversed the promotion of miR-inhibitor on cell apoptosis of TC (Figure 4(d)). These results displayed that miR-196a-2 targeted NRXN1 to stimulate cell proliferation and inhibit cell apoptosis of TC.

The article "miR-196a-2 Promotes Malignant Progression of Thyroid Carcinoma by Targeting NRXN1" was retracted in 2023. Reasons: signs of a paper mill; suspected computer-generated content; unreliable results or conclusions; concerns about the data.

## 4. Discussion

Accumulating reports manifested that miRNAs can serve as oncogenes or tumor suppressors, and aberrantly expressed miRNAs are often observed in varying tumors [12]. Currently, several miRNAs are identified to be molecular targets for cancer treatment. For example, miR-122-5p can inhibit cell proliferation and invasion of bile duct carcinoma by targeting ALDOA, showing its great potential as a molecule therapeutic target in the treatment of bile duct carcinoma [13]. miR-16-5p can regulate the expression of Smad3 to inhibit chordoma cell proliferation and metastasis, and it has also been proven to become a molecular therapeutic target for chordoma [14]. miR-196a-5p may play a key role in the epithelial-mesenchymal transition (EMT), invasion, and metastasis of colorectal cancer cells through targeting I*κ*B*α*, which has certain guiding significance for clinical treatment of human colorectal cancer [15]. Increased miR-196a facilitates cell proliferation of gastric cancer by p27 (kip1) suppression, which may be a therapeutic target for gastric cancer and further develop into a potentially prognostic factor [16]. miR-196a-2 is one of the subtypes of miR-196a located on chromosome 12 between HOXC 10 and HOXC 12, and there have been no relevant experiments validating that miR-196a-2 can regulate tumor progression so far [6]. Our results authenticated that miR-196a-2 was upregulated in TC cells. Silencing miR-196a-2 could inhibit cell proliferation and stimulate cell apoptosis of TC. These results proved the oncogenic role of miR-196a-2, which is a potentially therapeutic target for human TC in clinical. NRXN1 is a presynaptic neuron adhesion molecule that can interact with neurotrophic factors of inhibitory synapses in the brain to participate in the formation and maintenance of synapses [17, 18]. Several lines of evidence have illustrated that NRXN1 is a disease-causing gene related to mental illness, and knockdown of NRXN1 will result in a decrease in astrocytes produced by neural stem cells, thereby leading to autism and schizophrenia [19]. Through literature review, it is disclosed that there are few studies on role and mechanism of NRRX1 in cancer cells, and only a few studies have reported that NRRX1 is a gene related to cancer progression through bioinformatics methods. For instance, Sun et al. [20] disclosed that NRXN1 is associated with overall survival of patients with colorectal cancer via genome-wide methylation and expression profile identification, and NRXN1 may be a promising biomarker for colorectal cancer. Research by Yotsumoto et al. [21] manifested that NRXN1 can be a potentially novel target for antibody-drug conjugates in small-cell lung cancer. Based on bioinformatics methods, we found the binding relationship between miR-196a-2 and NRXN1 and verified that NRXN1 was lowly expressed in TC. Besides, it was found that miR-196a-2 downregulated NRXN1 and stimulated cell proliferation while repressed cell apoptosis of TC, which played an oncogenic role in TC.

The article "miR-196a-2 Promotes Malignant Progression of Thyroid Carcinoma by Targeting NRXN1" was retracted in 2023. Reasons: signs of a paper mill; suspected computer-generated content; unreliable results or conclusions; concerns about the data.

These observations collectively demonstrated for the first time that miR-196a-2 is upregulated in TC and can target and inhibit the expression of NRXN1, thereby promoting the malignant progression of TC. Hence, our study lays a theoretical foundation for miR-196a-2/NRXN1 to become a molecular therapeutic target for TC, generating novel insights and providing new strategies for TC. Nonetheless, specific mechanism of miR-196a-2 on TC needs to be further probed. Moreover, animal experiments *in vivo* need to be done to validate the oncogenic impact of miR-196a-2, thereby improving our investigation.

## Figures and Tables

**Figure 1:** miR-196a-2 is upregulated in TC. (a) qRT-PCR detected the expression of miR-196a-2 in HTori-3, TFC-133, TPC-1, and KTC-1. ^∗^*P* < 0.05.

**Figure 2:** Silencing miR-196a-2 inhibits cell proliferation and promotes cell apoptosis of TC. (a) The effect of miR-inhibitor on the expression of miR-196a-2 in FTC-133 cells detected by qRT-PCR; (b) the effect of silenced miR-196a-2 on the proliferation of FTC-133 cells detected by CCK-8; (c) the effect of silenced miR-196a-2 on the colony forming ability of FTC-133 cells detected by colony formation assay; (d) the effect of silenced miR-196a-2 on FTC-133 cell apoptosis observed by apoptosis assay; ^∗^*P* < 0.05.

**Figure 3:** NRXN1 is the direct target of miR-196a-2. (a) Binding sites between miR-196a-2 and NRXN1; (b, c) qRT-PCR and western blot detected the expression of NRXN1 in HTori-3, FTC-133, TPC-1, and KTC-1 cells; (d, e) the effect of silenced miR-196a-2 on the mRNA and protein expression of NRXN1 in FTC-133 cells detected by qRT-PCR and western blot; (f) the targeted binding relationship between miR-196a-2 and NRXN1 was predicted by bioinformatics analysis and identified by dual-luciferase reporter gene assay; ^∗^*P* < 0.05.

The article "miR-196a-2 Promotes Malignant Progression of Thyroid Carcinoma by Targeting NRXN1" was retracted in 2023. Reasons: signs of a paper mill; suspected computer-generated content; unreliable results or conclusions; concerns about the data.

**Figure 4:** miR-196a-2 regulates cell proliferation and cell apoptosis of TC by targeting NRXN1. (a) NRXN1 expression detected by qRT-PCR and western blot; (b) cell proliferative ability detected by CCK-8; (c) colony formative number detected by colony formation assay; (d) cell apoptosis detected by cell apoptosis assay. ^∗^*P* < 0.05.

**Table 1:** Primer sequences in qRT-PCR.

Target gene	Gene sequences
miR-196a-2	Forward: 5′-TCGGCAGGTAGGTAGTTTCTGT-3′
	Reverse: 5′-CTCAACTGGTGTCGTGGA-3′
NRXN1	Forward: 5′-TAAGTGGCCTCCTAATGACCG-3′
	Reverse: 5′-TCGCACCAATACGGCTTCTTT-3′
U6	Forward: 5′-GCTTCGGCAGCACATATACTAAAAT-3′
	Reverse: 5′-CGCTTCACGAATTTGCGTGTCAT-3′
GAPDH	Forward: 5′-GGAGCGAGATCCCTCCAAAAT-3′
	Reverse: 5′-GGCTGTTGTCATACTTCTCATGG-3′

## Data Availability

The data used to support the findings of this study are included within the article. The data and materials in the current study are available from the corresponding author on reasonable request.
